# Efficacy Analysis of DSA-Guided Bronchial Arterial Chemoembolization Interventional Therapy in Patients with Middle-Advanced Primary Bronchial Lung Cancer

**DOI:** 10.1155/2022/3722703

**Published:** 2022-03-23

**Authors:** Haili Cao, Shuqiang Jin, Bin Bai

**Affiliations:** Department of Interventional Radiology, The Second Affiliated Hospital of Harbin Medical University, Heilongjiang, Harbin 150086, China

## Abstract

**Objective:**

To investigate the clinical efficacy of digital subtraction angiography- (DSA-) guided bronchial arterial chemoembolization (BACE) in patients with primary bronchial lung cancer.

**Methods:**

A total of 178 patients with primary intermediate and advanced bronchial lung cancer admitted to our hospital from February 2019 to March 2020 were selected as the subjects, and they were divided into control group (84 cases) and observation group (94 cases) according to the different chemotherapy regimens adopted by the patients. The control group was treated with traditional perfusion chemotherapy, and the observation group was treated with DSA-guided BACE interventional therapy, treated for 4 cycles, and followed up until the end of June 2021. The short-term clinical efficacy, hemoptysis remission, and incidence of adverse reactions were compared between the two groups. The mortality and recurrence rates between the two groups from treatment to the end of follow-up were counted, and the quality of life after treatment and 1 year after treatment were compared.

**Results:**

The short-term remission rate (73.40% vs. 58.33%), disease control rate (93.62% vs. 84.52%), hemoptysis remission rate (75.00% vs. 41.51%), the quality of life after chemotherapy cycle (90.86 ± 2.55 vs. 78.04 ± 2.21), and the quality of life after 1 year of follow-up (85.68 ± 2.23 vs. 70.27 ± 1.72) in the observation group were significantly higher than those in the control group, and the difference was statistically significant (*P* < 0.05). The incidence of adverse reactions (9.57% vs. 20.24%), mortality (10.64% vs. 21.43%), and recurrence rate (11.70% vs. 27.38%) during the follow-up period in the observation group were significantly lower than those in control group, and the differences were statistically significant (*P* < 0.05).

**Conclusion:**

DSA-guided BACE interventional therapy for patients with primary middle-advanced bronchial lung cancer has significant efficacy, which can not only reduce the mortality and recurrence rate of patients but also improve the quality of life of patients, with fewer adverse reactions and high safety, which is worthy of promotion.

## 1. Introduction

Bronchial lung cancer is one of the common malignant tumors in China, which is common in elderly men, and its incidence and mortality are increasing year by year [1]. Its early symptoms are easily confused with other respiratory diseases. Therefore, most patients are already in the middle and late stages of the disease course at the time of diagnosis. At the time of diagnosis, the tumor has invaded large blood vessels, accompanied by obvious hilar and mediastinal lymph node metastasis, poor cardiopulmonary function, etc., losing the opportunity of surgical treatment [2]. For such patients, traditional radiotherapy, chemotherapy, or concurrent chemoradiotherapy can prolong survival and improve symptoms to a certain extent, but the overall efficacy is not satisfactory due to the heavier tumor burden in advanced patients, the effect of systemic chemotherapy and radiotherapy is not good, and the adverse reactions are obvious [3]. Bronchial artery chemoembolization (BACE) can block the blood supply of bronchial lung cancer lesions and cause ischemic necrosis. At the same time, the local effect of high-concentration chemotherapeutic drugs can significantly increase the concentration of chemotherapeutic drugs in the tumor area, significantly prolong the contact time with tumor tissue, and significantly improve the chemotherapy effect of tumor lesions and lymph node metastasis lesions, which improved the clinical efficacy significantly [4]. Due to the large bronchial anatomical variation, through the digital subtraction angiography (DSA) to show the direct blood supply artery of bronchial lung cancer is the key for the successful implementation of BACE [5]. At present, there are few comparative studies on DSA-guided BACE interventional therapy and conventional chemotherapy for lung cancer patients. This study retrospectively analyzed patients with primary middle-advanced bronchial lung cancer who received BACE treatment in the Interventional Therapy Department of our hospital and analyzed the clinical efficacy and safety of DSA-guided BACE interventional therapy for bronchial lung cancer patients.

## 2. Materials and Methods

### 2.1. Research Subjects

A total of 178 patients with primary middle-advanced bronchial lung cancer who received chemotherapy in our hospital from February 2019 to March 2020 were enrolled as the subjects, and they were followed up until the end of June 2021. Patients were divided into control group (84 cases) and observation group (94 cases) according to different chemotherapy methods. Inclusion criteria are as follows: (1) patients diagnosed as primary bronchial lung cancer by comprehensive diagnosis of X-ray, CT, MRI, PET-CT, bronchial arteriography, blood biochemical examination, and pathological tissue biopsy[6]; (2) patients in the middle and late stages of TNM staging who were unable or unwilling to undergo surgical resection; (3) no chemotherapy contraindications; (4) Karnofsky score > 70 points; (5) estimated survival time > 6 months; and (6) patients and their families understood the contents of this study and signed the written informed consent. Exclusion criteria are as follows: (1) patients using other chemotherapy or radiotherapy within a month; (2) patients complicated with other malignant tumors; (3) patients with a history of chest, bronchial, and lung surgery; (4) serum creatinine > 177 *μ*mol/L, Hb < 140 g/L, WBC < 3 × 10^12^/L; (5) partial or complete thrombosis of the pulmonary artery; (6) patients with a large amount of pleural fluid unable to lie down; (7) patients allergic to platinum drugs and contrast agents; (8) patients with severe osteoporosis; (9) patients with coagulopathy (platelets < 5 × 10^12^/L, prothrombin activity < 50%); and (10) patients with abnormal mental cognition. This study was reported and approved by the Medical Ethics Committee of our hospital.

### 2.2. Treatment Methods

The control group was given traditional infusion chemotherapy, and for patients with squamous cell carcinoma and small-cell lung cancer, 10-14 mg of mitomycin (specification: 2 mg × 5, Pfizer Pharmaceutical Co., Ltd., SFDA approval number: H20013213), 40~50 mg of adriamycin (specification: 10 mg × 5, Shenzhen Main Luck Pharmaceutical Co., Ltd., SFDA approval number: H44024359), and 50~80 mg of cisplatin (specification: 20 mg × 5, Qilu Pharmaceutical Co., Ltd., SFDA approval number: H20073653) were used. For patients with adenocarcinoma, 0.75 g~1 g of fluorouracil (specification: 0.25 g × 5, Beijing Zizhu Pharmaceutical Co., Ltd., SFDA approval number: H11020069), 40~50 mg of doxorubicin, and 300~400 mg of carboplatin (specification: 100 mg × 5, Qilu Pharmaceutical Co., Ltd., SFDA approval number: H20020180) were used.

Patients in the observation group underwent DSA-guided BACE interventional therapy (DSA, model: AXIOM Artis-dTA, Manufacturer: Siemens Co., Ltd., Germany). Seldinger puncture technique [7] was used to puncture the right femoral artery and inserted 5 Fr catheter sheath. Under C-arm fluoroscopy, guide wire and 5 Fr Cobra catheter were inserted along the catheter sheath to perform bronchial arteriography to determine the size, number, and staining of the tumor. Considering whether there were multiple bronchial arteries or other arteries supplying blood, then use microcatheter to select the target artery supplying blood to the tumor. About 5 ml of 1% lidocaine (specification: 5 ml × 5, Suicheng Pharmaceutical Co., Ltd., SFDA approval number: H41023668) was slowly injected through microcatheter. If no symptoms appeared, it was negative and BACE can be performed directly. Patients with weakness and numbness in both lower limbs were judged to be positive, indicating the possibility of spinal root artery emanating from bronchial artery. After that, three-dimensional (3D) DSA rotational angiography was performed. The total amount of contrast agent (ioversol injection, specification: 100 ml, 74.1 g/bottle, Jiangsu Hengrui Pharmaceutical Co., Ltd., SFDA approval number: H20143027) was 5 ml at a rate of 1 ml/s. High-pressure syringe 100 kPa (AngiomatIllumena, LF Company, USA) was used. The CT function of DSA was used for postprocessing 3D reconstruction to find the starting position of the spinal root artery, adjust the microcatheter, and perform BACE after avoiding the spinal root artery. After perfusion, embosphere embolization microsphere with appropriate size was chosen according to tumor size and blood supply (optional specification: 300-700 *μ*m in diameter (France Merit Medical Instrument Co., Ltd., China (importation) 2014 No. 3781181)), and it was mixed with an appropriate amount of contrast agent and injected via catheter under transmission for BACE. Angiography was performed while embolization was performed, and embolization was stopped when bronchial artery occlusion was shown and contrast agent retention appeared. The injection dose of microspheres was 0.5-3 mL, with an average of 2 mL. All patients were deprived of food and water before surgery, and skin preparation of the operative region was performed. Low-flow oxygen inhalation and ECG monitoring were continued during the operation, and stage analgesia was given according to the degree of pain. Urine retention, sensory disturbance, and limb movement were observed 2~4 hours after operation. Routine antiemetic, anti-inflammatory, hydration, and other adjuvant treatments were given. Every 3 weeks was a cycle. Imaging review was performed in each treatment cycle. If supply vessels and tumor staining had disappeared, no other medical intervention was required. If the tumor was still stained, the above interventional therapy was repeated and the efficacy was evaluated after 4 cycles of treatment. In the following six months, the patients were followed up monthly with imaging and laboratory examinations. After six months, the patients were followed up once every three months.

### 2.3. Observation Indicators and Evaluation Criteria of Efficacy

(1) The recent clinical efficacy of the two groups was compared according to the tumor remission criteria formulated by the Union for International Cancer Control (UICC) [8]: the volume of the tumor was the product of the two largest mutually perpendicular diameters of the tumor. Remission criteria were as follows: ① complete remission (CR): the tumor disappeared completely, and no tumor was found in the original site by palpation and visual examination; ② partial remission (PR): the measured tumor parameters were reduced by 50% or more, and no new lesions appeared; ③ stable disease (SD): the tumor reduced by less than 50% or increased by less than 25%; ④ progression disease (PD): the measured tumor parameters increased by more than 25% or new lesions appeared. A 50% reduction in tumor size or significant relief of symptoms was considered effective. Objective response rate (ORR): it is the proportion of patients whose tumors had shrunk to a certain extent and maintained for a certain period of time, ORR = (CR + PR)/total number of cases × 100%, and disease control rate = (CR + PR + SD)/total number of cases × 100%. (2) The relief of hemoptysis was compared between the two groups. The evaluation principles for the relief of hemoptysis included are as follows: ① hemoptysis was stopped immediately within 24 hours after operation, and no special medical treatment was needed to stop the bleeding; ② hemoptysis stopped immediately, only a small amount of blood in the sputum can be treated by medical treatment to stop the bleeding; ③ hemoptysis was reduced by 50% or more than before. (3) The incidence of adverse reactions was compared between the two groups. (4) The mortality rate and recurrence rate of patients in the two groups from treatment to the end of follow-up were counted, and the recurrence rate was assessed according to the clinical standards of Chinese Medical Association guidelines for clinical diagnosis and treatment of lung cancer (2019 edition) [8]. (5) The quality of life of patients after completing the chemotherapy cycle and 1 year after treatment was compared between the two groups. The Chinese version of WHO Quality of Life-BREF (WHOQOL-BREF) was used for evaluation [9], with a total of 26 questions and a total score of 100 points. The higher the score, the better the quality of life

### 2.4. Statistical Analysis

Statistical analysis was performed using the SPSS 22.0 software. The measurement data conformed to the normal distribution was represented by $\bar{x}\pm s$, the comparison between the two groups was performed by independent sample *t*−test, and the comparison among multiple groups was performed by one-way ANOVA; the count data was represented by *n* (%), and comparison between groups was performed by *χ*^2^ test; *P* < 0.05 was considered statistically significant.

## 3. Results

### 3.1. Comparison of General Clinical Data

There was no statistically significant difference in gender, age, pathological type, TNM stage, tumor site, and KPS score between the two groups of patients (*P* > 0.05), and they were comparable (see Table 1 for details).

### 3.2. Comparison of the Short-Term Clinical Efficacy of the Two Groups of Patients

In the control group, there were 84 patients, including 12 cases of CR (14.29%), 37 cases of PR (44.05%), 22 cases of SD (26.19%), 13 cases of PD (15.48%), and the ORR was 58.33% (49/84); the disease control rate was 84.52% (71/84). Among the 94 patients in the observation group, there were 17 cases of CR (18.09%), 52 cases of PR (55.32%), 19 cases of SD (20.21%), and 6 cases of PD (6.38%), ORR was 73.40% (69/94), and the disease control rate was 93.62% (88/94). The difference in ORR and disease control rate between the two groups was statistically significant (*P* < 0.05), and the specific data are shown in Table 2.

### 3.3. Comparison of the Remission Rate of Hemoptysis between the Two Groups

In the control group, 53 patients had mild to moderate hemoptysis, and 22 patients were relieved after treatment, with a remission rate of 41.51%. In the observation group, 64 patients had mild to moderate hemoptysis, and 48 patients had their symptoms relieved after treatment, with a remission rate of 75.00%. The remission rate of hemoptysis was compared between the two groups, and the difference was statistically significant (*χ*^2^ = 13.530, *P* < 0.001), as shown in Figure 1. In this study, there were 5 patients with severe hemoptysis in the control group. There were 3 patients with severe hemoptysis in the observation group. All 8 patients died after severe hemoptysis.

### 3.4. Comparison of the Incidence of Adverse Reactions between the Two Groups

Adverse symptoms such as nausea, vomiting, anorexia, and fever caused by chemotherapy can be alleviated by oral medication. In both groups, severe adverse reactions such as spinal cord injury occurred. In the observation group, there were 2 cases of mild chest pain on the side of embolism, and the incidence of adverse reactions was 9.57% (9/94). The incidence of adverse reactions in the control group was 20.24% (17/84), and the difference between the two groups was statistically significant (*P* < 0.05) (see Table 3 for specific data).

### 3.5. Mortality and Recurrence Rate during the Follow-Up Period of the Two Groups of Patients

All patients enrolled in this study were followed up to the end of June 2021, with the longest follow-up of 25 months and the shortest follow-up of 12 months, with an average follow-up of 17.68 ± 3.25 months. During the follow-up period, the mortality and recurrence rates in the observation group were significantly lower than those in the control group, with statistical significance (*P* < 0.05), as shown in Table 4.

### 3.6. Comparison of Quality of Life between the Two Groups of Patients

The comparison of changes in quality of life between the two groups after completing the chemotherapy cycle and after 1-year follow-up is shown in Table 5. Quality of life score of the observation group was significantly higher than the control group, and the difference was statistically significant (*P* < 0.05).

## 4. Discussion

Bronchial lung cancer is a malignant tumor originating from the endobronchial epithelial cells. Under the influence of the environment and the increasing number of long-term heavy smokers, the incidence and mortality of lung cancer have increased significantly in China. The onset of the disease is insidious, and the early clinical symptoms are not obvious. When patients present clinical symptoms, they have reached the middle and late stages, and the tumor has involved adjacent structures or distant metastasis, thus losing the best treatment opportunity for surgical resection. Generally, intravenous chemotherapy, radiotherapy, and molecular-targeted therapy are the main treatment methods for middle-advanced lung cancer. However, there are many side effects of intravenous chemotherapy and radiotherapy, and some patients cannot tolerate them, so the effective rate is not satisfactory [10]. Targeted therapy is expensive, requires gene locus detection, and is not suitable for all lung cancer patients.

With the development of interventional radiology, perfusion chemotherapy for tumor supplying artery emerged, and the arterial perfusion chemotherapy for middle-advanced lung cancer has been gradually recognized and accepted. Clinical studies have shown that the nutrition of lung cancer does not come from the blood supply of pulmonary artery, but mainly from the bronchial artery [11]. On the one hand, transbronchial artery infusion of chemotherapeutic drugs improves the local drug concentration of the tumor due to organ targeting and first-pass effect, while the peripheral drug concentration does not increase. Compared with intravenous chemotherapy, it not only improves the efficacy but also reduces the systemic adverse reactions and damage to normal tissues [12]. On the other hand, bronchial artery embolization can not only prolong the residence time of chemotherapy drugs in tumor tissues and enhance the therapeutic effect of chemotherapy drugs but also effectively block the blood-supply vessels of tumor tissues, resulting in ischemia, necrosis, and shrinkage of tumor tissues [13].

In this study, patients in the observation group underwent DSA-guided bronchial arterial infusion chemotherapy, and the short-term tumor remission rate was as high as 73.40%, and the short-term disease control rate was as high as 93.62%. During 1-2 years of follow-up after operation, the mortality and recurrence rates of patients were significantly lower than those of the control group. Other studies have shown [14] that after 1 year of interventional therapy, the survival rate of patients was 58.92%, which may be related to the success rate of BACE. In this study, 1% lidocaine was injected in the DSA operating room to determine whether the spinal root artery, bronchial artery, and intercostal artery had common trunk and the location of common trunk, and then, BACE was performed, which improved the success rate of BACE and reduced the incidence of spinal injury.

Li et al. [15] believe that BACE for advanced lung cancer with hemoptysis is safe, effective, and tolerable. In this study, the incidence of adverse reactions in the observation group was significantly lower than that in the control group. In this study, there were 16 cases of severe hemoptysis in the control group and the observation group. These patients all died after severe hemoptysis. Therefore, this study counts the remission rate of hemoptysis in patients with mild to moderate hemoptysis. The remission rate of hemoptysis in the observation group was higher than that in the control group. Comparing the changes in the quality of life of the two groups of patients after completing the chemotherapy cycle and after 1 year of follow-up, the results showed that the quality of life score of the observation group was significantly higher than that of the control group. Previous studies have shown that bronchial arterial chemoembolization is safe and effective in the treatment of refractory and relapsed non-small-cell lung cancer and can be used as a good choice for the clinical treatment of refractory and relapsed non-small-cell lung cancer [16].

In summary, DSA-guided BACE interventional therapy for patients with primary middle-advanced bronchial lung cancer can improve the success rate of BACE and ensure the effect of interventional therapy for lung cancer. It can not only reduce the mortality and recurrence rate of patients and improve the quality of life of patients, but also have fewer adverse reactions and high safety, which is worth of promotion. This research still has certain flaws. The clinical application of chemotherapy has certain uncontrollable factors on the research results. And the study is a retrospective study. This study can provide certain guiding significance for the follow-up of large-sample, multi-center clinical research.

## Figures and Tables

**Figure 1:** Comparison of the remission rate of hemoptysis between the two groups.

**Table 1:** Comparison of basic clinical data between the two groups.

Indicator	Control group (*n* = 84)	Observation group (*n* = 94)	*χ* ^2^/*t* value	*P* value
Gender (male/female) (*n*)	50/34	52/42	0.417	0.519
Age(years)	55.07 ± 9.81	54.34 ± 11.68	0.451	0.652
Pathological classification (*n*)			0.123	0.940
Adenocarcinoma	46	50		
Squamous cell carcinoma	11	14		
Small-cell lung cancer	27	30		
TNM staging (*n*)			0.153	0.926
IIIa	16	18		
IIIb	38	40		
IV	30	36		
Tumor site (*n*)			0.395	0.941
Left upper lobe	17	16		
Left lower lobe	12	14		
Right upper lobe	35	39		
Right lower lobe	20	25		
KPS score	78.80 ± 6.10	79.11 ± 5.77	0.342	0.733

**Table 2:** Comparison of short-term clinical efficacy between the two groups of patients (*n*, %).

Group	CR	PR	SD	PD	ORR	Disease control rate
Control group (*n* = 84)	12 (14.29)	37 (44.05)	22 (26.19)	13 (15.48)	49 (58.33)	71 (84.52)
Observation group (*n* = 94)	17 (18.09)	52 (55.32)	19 (20.21)	6 (6.38)	69 (73.40)	88 (93.62)
*χ* ^2^ value	0.470	2.254	0.894	3.847	4.509	3.900
*P* value	0.493	0.133	0.344	0.05	0.034	0.048

**Table 3:** Comparison of the incidence of adverse reactions between the two groups (*n*, %).

Adverse reactions	Control group (*n* = 84)	Observation group (*n* = 94)	*χ* ^2^ value	*P* value
Nausea and vomiting	8 (9.52)	5 (5.32)		
Anorexia	3 (3.57)	4 (4.25)		
Fever	2 (2.38)	4 (4.25)		
Chest pain	6 (7.14)	2 (2.13)		
Myocardial damage	2 (2.38)	1 (1.06)		
Decreased hemoglobin	5 (5.95)	2 (2.13)		
Total incidence rate	17 (20.24)	9 (9.57)	4.076	0.043

**Table 4:** Mortality and recurrence rate during the follow-up period of the two groups of patients (*n*, %).

Group	Number of cases	Death	Recurrence
Control group	84	18 (21.43)	23 (27.38)
Observation group	94	10 (10.64)	11 (11.70)
*χ* ^2^ value		3.896	7.057
*P* value		0.048	0.008

**Table 5:** Comparison of WHOQOL-BREF scores between the two groups.

Group	Number of cases	After the end of the chemotherapy cycle	After 1 year of follow-up
Control group	84	78.04 ± 2.21	70.27 ± 1.72
Observation group	94	90.86 ± 2.55	85.68 ± 2.23
*t* value		35.621	51.232
*P* value		<0.01	<0.01

## Data Availability

The labeled dataset used to support the findings of this study are available from the corresponding author upon request.
